# Modeling Dynamics of *Culex pipiens* Complex Populations and Assessing Abatement Strategies for West Nile Virus

This article has been retracted.

**DOI:** 10.1371/journal.pone.0108452

**Published:** 2014-09-30

**Authors:** Kasia A. Pawelek, Patrick Niehaus, Cristian Salmeron, Elizabeth J. Hager, Gregg J. Hunt

**Affiliations:** 1 Department of Mathematics and Computational Science, University of South Carolina Beaufort, Bluffton, South Carolina, United States of America; 2 Beaufort County Mosquito Control, Beaufort, South Carolina, United States of America; University of Texas Medical Branch, United States of America

## Abstract

The primary mosquito species associated with underground stormwater systems in the United States are the *Culex pipiens* complex species. This group represents important vectors of West Nile virus (WNV) throughout regions of the continental U.S. In this study, we designed a mathematical model and compared it with surveillance data for the *Cx. pipiens* complex collected in Beaufort County, South Carolina. Based on the best fit of the model to the data, we estimated parameters associated with the effectiveness of public health insecticide (adulticide) treatments (primarily pyrethrin products) as well as the birth, maturation, and death rates of immature and adult *Cx. pipiens* complex mosquitoes. We used these estimates for modeling the spread of WNV to obtain more reliable disease outbreak predictions and performed numerical simulations to test various mosquito abatement strategies. We demonstrated that insecticide treatments produced significant reductions in the *Cx. pipiens* complex populations. However, abatement efforts were effective for approximately one day and the vector mosquitoes rebounded until the next treatment. These results suggest that frequent insecticide applications are necessary to control these mosquitoes. We derived the basic reproductive number (ℜ_0_) to predict the conditions under which disease outbreaks are likely to occur and to evaluate mosquito abatement strategies. We concluded that enhancing the mosquito death rate results in lower values of ℜ_0_, and if ℜ_0_<1, then an epidemic will not occur. Our modeling results provide insights about control strategies of the vector populations and, consequently, a potential decrease in the risk of a WNV outbreak.

## Introduction

West Nile virus (WNV) is a vector-borne enzootic pathogen amid a bird-mosquito-bird cycle throughout small to large regional areas, with humans and horses as incidental hosts [1]–[3]. A portion of mosquitoes potentially associated with WNV may rest and/or breed in underground stormwater systems, such as catch basins. These stormwater structures are engineered to drain excess rain water from streets, parking lots, and other non-pervious areas [4], [5]. Mosquitoes may develop in large numbers in the nutrient-rich standing water among the catch basins and adjacent pipes. The most important mosquito species adopting this underground habitat in the United States is the *Culex pipiens* complex (*Cx. pipiens* Linnaeus, *Cx. quinquefasciatus* Say, and/or hybrids), primary vectors for WNV in the northern and southern regions, including Beaufort County, South Carolina [6].

Forty-eight states reported at least 39,000 human cases of WNV infection with 1,663 fatalities as a major health concern in the U.S. during 1999–2013 [7], [8]. In SC, 73 human cases of WNV, including 5 deaths, were confirmed from 2002–2013 [9]. Anyone living in or visiting an area where WNV is prevalent is at risk of becoming infected. [1]. In humans, WNV infection may be asymptomatic or may cause febrile illness, encephalitis, or meningitis [1], [10]. Although the majority (about 80%) of WNV-infected people are asymptomatic [1], adults at least 50 years of age have the greatest risk of developing the more severe symptoms of WNV upon infection [11]. Approximately 20% of the people infected with WNV will show flu-like symptoms whereas less than 1% of infected individuals will develop neurologic illness causing severe or life-threatening symptoms [1].

Public health insecticides (for immature and adult mosquitoes) and source reduction (elimination of mosquito breeding sites) represent important strategies to reduce the risk of WNV outbreaks throughout the U.S. [12]. The application of larvicides and adulticides must be conducted in a timely manner. Other risk-reducing approaches include the use of insect repellents and protective clothing as well as avoidance of peak mosquito feeding hours [1].

Public health plans developed before and during a disease epidemic are typically influenced by previous outbreaks. Further, mathematical models are needed to test abatement strategies based on current and past epidemics. For example, mathematical models represented an important tool in preparation for an influenza outbreak [13], [14]. A number of models have also been developed to study within-host dynamics of virus infections (for instance, [15], [16]). Susceptible, Exposed, Infected, Recovered (SIR/SEIR) models have been studied [17], [18] and various mathematical models have been developed to study the spread of WNV [19]–[24]. Also, models have examined insecticide treatments to reduce mosquito and Triatomine bug populations, such as during malaria [25] and Chagas disease outbreaks, respectively [26], [27]. However, only a few models have studied the abatement strategies used for WNV intervention [28], [29]. Mathematical models for WNV transmission and calculations of the basic reproductive ratio, which is used to predict disease outbreaks and evaluate abatement strategies, have been compared to each other [21]. The study concluded that model assumptions are the key features when finding the basic reproductive ratio and varying assumptions may lead to contradictory results [21]. The feeding preferences of *Cx. pipiens* were evaluated for preferred and alternative bird species [22]. The study suggested that inclination of mosquitoes to feed on the American robin (*Turdus migratorius* Linnaeus) was the key parameter influencing the timing of the WNV infection peak [22]. Mosquito reduction strategies and personal protection were evaluated using a single-season deterministic model during a WNV outbreak [28]. The analysis of equilibria was conducted to determine the conditions for the WNV persistence [28]. None of the aforementioned articles examined the insecticide effectiveness based on surveillance data and simultaneously estimate the disease burden during a WNV outbreak, which we investigated in this study.

We developed a mathematical model established on previous modeling techniques [28], [30] and compared the model with *Cx. pipiens* complex surveillance data to estimate the parameters associated with treatment effectiveness, as well as mosquito birth, maturation, and death rates. We employed the obtained estimates in an epidemiological model with various severity stages of the disease to test the mosquito abatement strategies during a WNV outbreak. This allowed us to obtain more precise predictions, which are crucial to develop and implement control strategies during a disease outbreak. Further, we obtained possible disease burden estimates by organizing the human population into various disease severity stages. These scenarios could be essential when various control strategies are used, such as drug administration, during limited medication supply and/or resistance.

## Materials and Methods

### Study area

Beaufort County is located within the Lower Coastal Plain in the southern portion of SC. The topography is generally low and flat with vast wetlands, including tidal salt and brackish waters as well as bottomland hardwood swamps [31]. Beaufort County consists of 923 square miles (576 square miles for land and 347 square miles for water) with about 168,000 residents [32]. Various habitats for birds, animals, mosquitoes, and other insects are located throughout Beaufort County [31]. Approximately 39.7% of the Beaufort County population consists of adults who are 50 years and older [33]. Sun City Hilton Head (located near the Town of Bluffton in Beaufort County) is the largest senior adult community in SC, with over 13,000 residents [34].

### Study sites

The study sites consisted of the Sams Point neighborhood on Ladys Island (Figure 1) and the Battery Point neighborhood on Port Royal Island (Figure 2). The GPS coordinates were 32.423717–80.644145 and 32.422526–80.711176, respectively. These neighborhoods share similarities: urban residential communities, commercial properties, underground stormwater systems, roadside ditches, moderate to large tree canopies, navigable waterways, pest and/or vector mosquitoes, and feral birds.

**Figure 1:** Aerial view of Sams Point neighborhood on Ladys Island, Beaufort County, SC depicting the location of the mosquito collection trap and various underground stormwater catch basins.

**Figure 2:** Aerial view of Battery Point neighborhood on Port Royal Island, Beaufort County, SC depicting the location of the mosquito collection trap and various underground stormwater catch basins.

### Mosquito collections

As part of the surveillance program, Beaufort County Mosquito Control (BCMC) operated 20 strategically located mosquito traps (which included the two study sites) within the underground stormwater systems throughout Beaufort County. Encephalitis Vector Survey (EVS) traps (BioQuip Products, San Dominguez, CA) were used for the weekly collections. The traps were suspended underground below the catch basin lids and were operated for about 24 continuous hours each week. Each EVS trap included a blue LED light bulb and CO2 (approximately 3 pounds of dry ice) as attractants whereas a down-draft fan captured the mosquitoes into a collection net. From 2006 to 2012, weekly collections were identified to male and female species using a stereo microscope. We evaluated the *Cx. pipiens* complex for modeling because the mosquito species are the most abundant vectors for WNV in the study area.

### Public health insecticide treatments

As part of the integrated mosquito management (IMM) program, BCMC used three abatement strategies (as needed) in 2006–2012 to control immature and adult pest and/or vector mosquitoes throughout Beaufort County, including the two study sites (except aerial spraying). For the first strategy, BCMC applied a larvicide (Altosid XR briquets) to about 20,000 catch basins, including those stormwater structures at Sams Point and Battery Point neighborhoods, at the beginning of each mosquito season. The application rate was one briquet per catch basin. This product was used to control mosquito breeding and was effective for up to 5 months (according to the manufacturer label) or longer depending on the frequency of rain events. BCMC used mapping software (ESRI ArcGIS ArcMap 10.1, Redlands, CA) to geocode this large inventory of catch basins. The treatment of aboveground breeding sites for the *Cx. pipiens* complex is mostly nonexistent because this type of breeding occurs among various water-holding containers (bird baths, waste tires, etc.) on private properties. For the second strategy, BCMC operated up to 7 spray trucks using various Ultra-Low Volume (ULV) adulticiding products during the 7-year-long study (Table 1). Before the start of each mosquito season, BCMC evaluated the efficacy rate (via 24-hour bioassays) of the adulticiding product selected for use. The efficacy rates ranged from 91–100% (Table 1). These ground-dispersed products are effective as contact insecticides during the night in which most of the active ingredients break down within an hour after sunlight exposure. For the third strategy, BCMC operated a fixed wing aircraft using another adulticide, Anvil 10+10 ULV (0.48 ounces per acre with a 90% efficacy rate), during mostly sunrise. However, aerial spraying did not occur at the two study sites because beehives and/or fish-bearing waters existed at both sites.

**Table 1:** Public health insecticides applied from spray trucks to control adult mosquitoes throughout Beaufort County, SC (including the two study sites) during 2006–2012.

Year	Public Health	Application Rate	Efficacy Rate (%)*
	Insecticide	(ounces per acre)	
2006	Aqua-Reslin	0.69	100
2007	Aqua-Reslin	0.69	100
2008	Aqualuer 20-20	0.55	91
2009	Aqualuer 20-20	0.55	91
2010	Zenivex E20	0.57	94
2011	Evoluer 30-30	0.83	93
2012	Evoluer 30-30	0.83	93

*After 24-hour bioassays.

The mosquito surveillance data was examined to determine the relationships between the *Cx. pipiens* complex populations and the effects of the insecticide treatments during June-September when the highest average temperature and rainfall data were typically recorded (temperature data from [35]).

### Ethics statement

A permit to conduct the study within Beaufort County was not required because the underground stormwater systems (including catch basins) are owned and maintained by several governmental entities, such as SC Department of Transportation, Beaufort County, and/or various municipalities. Specific permission was not required to conduct surveillance of mosquitoes collected at the various catch basins. However, the Director of BCMC coordinated activities with the Director of Beaufort County Public Works (who is responsible for the drainage infrastructure systems). BCMC applicators possess SC Non-Commercial Applicator Licenses as certified by Clemson University Department of Pesticide Regulation. County Council of Beaufort County has approved an annual budget for BCMC since 1974 and continues to endorse the control of mosquitoes and mosquito-borne diseases throughout its political boundary. Our field study did not involve endangered or protected species.

### Mathematical model

Mathematical modeling is frequently used to study the dynamics of vector populations and disease outbreaks [17]–[30], [36]. In this study, we designed a mathematical model based on Ordinary Differential Equations (model equations are listed in the Appendix S1 in File S1) to predict larval and adult mosquito populations and study the potential spread of WNV among birds and humans under various insecticide application scenarios and parameter estimates.

In the model, similar to [30], [37], we assume that WNV transmission is dependent on the abundance of bird reservoirs and humans. The model consists of three populations: bird reservoirs, potential *Cx. pipiens* complex vectors, and human populations, which are organized into subpopulations based on the development and/or severity of WNV infection. Naïve adult *Cx. pipiens* complex mosquitoes (*M_S_*), exposed (*M_E_*), and infectious (*M_I_*) adult mosquitoes lay eggs and, afterward, larvae (*L*) are born at the rate *b*. Larvae (*L*) originating from non-infected, exposed, and infectious mosquitoes mature to become susceptible adult mosquitoes (*M_S_*) at the rate *m*. The natural death rates of larvae and three populations of adult mosquitoes are denoted by *δ_L_* and *δ_M_*, respectively. The naïve, exposed, and infectious mosquitoes have the same natural death rate (*δ_M_*) because it is difficult to determine the cause of death.

We take the average number of mosquito bites on both birds and humans to be dependent on the total sizes of these populations because mosquitoes feed on birds and humans. The term *βα_H_M_I_H_S_*/*N_Total_* represents the rate of reservoir-frequency dependent infection when an infectious mosquito (*M_I_*) takes a blood meal from a susceptible human (*H_S_*), in which *β* is the average biting rate per day, *α_H_* is the probability of virus transmission to human per infectious bite, and *N_Total_* is the total blood supply of the entire populations of humans *N_H_* = *H_S_*+*H_E_*+*H_F_*+*H_N_*+*R*, and birds *N_B_* = *B_S_*+*B_I_*+*B_R_*. In the rate of infection, the fraction of mosquito bites on susceptible humans is represented by the ratio of susceptible humans to the total populations of humans and birds, *H_S_*/*N_Total_*. The disease incubation period in humans is denoted by *1/δ_E_*. After *1/δ_E_* days, a portion of the population (*κ*) develops WNV neuroinvasive disease (acute flaccid paralysis, encephalitis, or meningitis) (*H_N_*). Another segment of the population (*γ*) is asymptomatic/recovered (*R*) and the remaining portion of the infected individuals (*1-κ-γ*) develops WNV fever (*H_F_*). We did not distinguish between asymptomatic and recovered individuals because both populations do not exhibit any disease symptoms. After *1/δ_E_* days, all of the individuals with WNV fever (*H_F_*) recover and they are reclassified in the recovered category (*R*), because it is uncommon to die from the WNV fever [10]. Due to the severity of the neuroinvasive disease, a fraction of these individuals (*ω*) will die after *1/δ_N_* days and they are repositioned in the deceased individual category (*D*).

Infected mosquitoes (*M_I_*) may transmit the disease to susceptible birds (*B_S_*) at the reservoir-frequency dependent rate *βα_B_M_I_B_S_*/*N_Total_*, where *α_B_* is the probability of virus transmission to a bird per infectious bite and fraction of mosquito bites on susceptible birds is represented by the ratio of susceptible birds to the total populations of humans and birds, *B_S_*/*N_Total_*. Due to the severity of the disease, a fraction of infected birds (*σ*) will die after 1/δB days and the rest of the birds (*1-σ*) will recover. The infected, recovered, and dead birds due to the infection with WNV categories are represented by *B_I_*, *B_R_*, and *B_D_*, respectively. For simplicity, the birth or immigration of susceptible birds is represented by the recruitment rate *Λ*. Recruitment of infected birds could be taken into consideration by assuming that the fraction of the recruited birds *fΛ* is infected and the remaining proportion *(1-f)Λ* is susceptible. The natural death rates of birds in all categories are represented by *τ*.

Finally, susceptible mosquitoes (*M_S_*) become exposed to the infection at the reservoir-frequency dependent rate *βα_M_M_S_B_I_*/*N_Total_* when these insects bite an infected bird (*B_I_*), where *α_M_* is the probability of virus transmission to a mosquito per infectious bite and the fraction of mosquito bites on infected birds is represented by the ratio of infected birds to the total populations of humans and birds, *B_I_*/*N_Total_*. The viral incubation rate in mosquitoes is denoted by *η*. We omitted the natural death, birth, and recruitment rates of human populations because of the short duration of the considered disease outbreak (one-season) and for model simplicity.

In the model, the population of adult mosquitoes (*M_S_, M_E_*, and *M_I_*) is decreased by insecticide interventions. The insecticide treatment is represented by the step function *S(t)*, which is equal to the insecticide treatment effectiveness (*s*) for the duration of its activity (*α*) and 0 when the treatment is inactive (insecticide treatment function is listed in the Appendix S1 in File S1). In this study, we investigate the effect of varying treatment effectiveness and frequency of its applications.

The schematic representation of the model including the spread of WNV among the populations is given in Figure 3, whereas model variables and parameters are listed in Tables 2 and 3, respectively. The model equations are shown in the Appendix S1 in File S1.

**Figure 3:** Schematic representation of the model. Model equations, variables, and parameters are given in the Appendix S1 in File S1, Tables 2 and 3, respectively.

**Table 2:** Definitions of variables used in the model.

Variable	Definition	Initial Condition
*L*	Female larval mosquito density	*L_0_ = L(0) = 1,000*
*M_S_*	Susceptible female adult mosquito density	*M_0_ = M_S_(0) = 1,000*
*M_E_*	Exposed female adult mosquito density	*M_E_(0) = 0*
*M_I_*	Infectious female adult mosquito density	*M_I_(0) = 1/M_0_*
*B_S_*	Susceptible bird density	*B_0_ = B_S_(0) = 1,000*
*B_I_*	Infectious bird density	*B_I_(0) = 0*
*B_R_*	Recovered bird density	*B_R_(0) = 0*
*B_D_*	Dead birds due to the infection with WNV density	*B_D_(0) = 0*
*H_S_*	Number of susceptible humans	*N = H_S_(0) = 1,000*
*H_E_*	Number of exposed humans	*H_E_(0) = 0*
*H_F_*	Number of humans with WNV fever	*H_F_(0) = 0*
*H_N_*	Number of humans with neuroinvasive disease	*H_N_(0) = 0*
*R*	Number of recovered humans	*R(0) = 0*
*D*	Number of dead humans	*D(0) = 0*

Sensitivity analysis of initial conditions is illustrated in Figure S3 in File S1.

**Table 3:** Parameter definitions, values, and references.

Symbol	Definition, Units	Range, Reference	Value, Reference
*s*	Treatment effectiveness, Day^−1^	0–1	fitted
*α*	Treatment duration, Days	0–1	1^I^
*b*	Birth rate, Larvae Day^−1^ Adults^−1^	0.02–0.15, calculated^II^	fitted
*δ_M_*	Natural death rate of adult mosquitoes, Day^−1^	0.02–0.07, [54], [55]	fitted
*δ_L_*	Natural death rate of larvae, Day^−1^	0.01–0.06, [54], [55]	fitted
*m*	Maturation rate of larvae, Adults Larvae^−1^ Day^−1^	0.05–0.09, [37], [56], [57]	fitted
*β*	Biting rate per day	1–5III	mean
*α_B_*	Probability of virus transmission to bird per infectious bite	0.27–1.00, [18], [39], [58]–[60]	mean
*α_M_*	Probability of virus transmission to mosquito per infectious bite	0.23–1.00, [18], [28], [38], [39], [59], [61]	mean
*α_H_*	Probability of virus transmission to human per infectious bite	-	0.88, [28]
*1/δ_B_*	Duration of viremia in birds, Days	3.8–6.0^IV^, [43]	4.5^IV^, [43]
*1/δ_E_*	Incubation period for humans, Days	2–6	mean
*1/δ_F_*	Duration of the WN fever, Days	-	14, [28]
*1/δ_N_*	Duration of the neuroinvasive disease, Days	33–42, [62]	mean
*κ*	Fraction of the human population that can develop neuroinvasive disease	-	<0.01^V^, [1]
*γ*	Fraction of the human population that is asymptomatic	0.7–0.8, [1]	mean
*ω*	Fraction of the human population with the neuroinvasive disease dying from the disease	-	0.1, [1]
*σ*	Fraction of the WNV-infected bird population dying from the disease	0.5–1.0^IV^, [43]	0.72^IV^, [43]
*η*	Virus incubation in mosquitoes, Day^−1^	0.09–0.12, [63]	0.1, [63]
*Λ*	Recruitment rate of susceptible birds, Birds Day^−1^	-	1.5^VI^
*τ*	Natural death rate of birds, Day^−1^	0.001–0.002, [22], [37], [64]	0.0015, [22], [37], [64]

I Value based on BCMC field observations and discussions.

II The lower and upper bounds for the birth rate were calculated based on the steady state, *δ_M_(m+δ_L_)/m* of the model without the infection, and the upper and lower bounds of the parameters utilized in the formula.

III It was estimated that *Culex quinquefasciatus* has 1–5 gonotrophic cycles [65], which are directly related to the number of blood meals taken by the mosquito [66]. We have also varied the values of mosquito biting rate in Figure 8 and Figure S4 in File S1.

IV Values taken from [43] for the following bird species: blue jay, house finch, American crow, house sparrow, and fish crow, which are mainly tested by SCDHEC [67].

V In simulations we assume κ = 0.01 to account for the worst case disease outbreak scenario.

VI The bird recruitment rate was calculated based on the steady state, Λ = *τB*_0_ of the model without the infection.

### Basic reproductive number

We determined the basic reproductive number (ℜ_0_) for the model (Appendix S2 in File S1). The threshold ℜ_0_ is one of the most influential tools developed to analyze and interpret models [38]–[41]. Basic reproductive ratio (ℜ_0_) is described as the average number of new infections caused by a single case in a fully susceptible population. If ℜ_0_>1, then an epidemic will arise whereas if ℜ_0_<1, then an epidemic will not occur. The Next Generation Method [42] was employed to determine ℜ_0_ (see Appendix S2 in File S1 for derivation). The dependence of ℜ_0_ on the mosquito death rate (*δ_M_*) and the mosquito biting rate per day (*β*) was investigated in this study.

### Data fitting and parameter values

We compared the model with the number of *Cx. pipiens* complex mosquitoes collected in traps located at the Sams Point and Battery Pont neighborhoods from 2006 to 2012 (Figure 4 and Table 4). We considered the months of June-September separately for each year and the corresponding insecticide applications.

**Figure 4:** Model comparison with mosquito surveillance data. Model predictions of adult mosquito populations (blue lines) based on the best-fit to *Culex pipiens* complex surveillance data collected during the summer months at the Sams Point and Batter Pont trap locations (blue dots) during 2006–2012. The best-fit parameters estimates are listed in Table 4.

**Table 4:** Best fit parameter values to the *Culex pipiens* complex surveillance data.

	Location: Sams Point					
Year	*δ_M_*	*δ_L_*	*b*	*m*	*s*	*p*
2006	3.6×10^−2^	1.6×10^−2^	3.8×10^−2^	9.0×10^−2^	7.0×10^−1^	3.4×10^−2^
2007	2.1×10^−2^	6.0×10^−2^	7.7×10^−2^	5.0×10^−2^	1.0×10^0^	6.6×10^−2^
2008	2.2×10^−2^	4.5×10^−2^	3.0×10^−2^	5.0×10^−2^	7.0×10^−1^	3.9×10^−2^
2009	3.9×10^−2^	1.0×10^−2^	7.4×10^−2^	7.8×10^−2^	7.1×10^−1^	2.4×10^−2^
2010	3.1×10^−2^	1.0×10^−2^	8.7×10^−2^	9.0×10^−2^	7.0×10^−1^	5.0×10^−3^
2011	7.0×10^−2^	1.9×10^−2^	1.5×10^−1^	9.0×10^−2^	8.3×10^−1^	7.3×10^−4^
2012	5.2×10^−2^	3.0×10^−2^	3.0×10^−2^	6.4×10^−2^	7.2×10^−1^	1.4×10^−2^
**Average**	3.9×10^−2^	2.7×10^−2^	6.9×10^−2^	7.3×10^−2^	7.7×10^−1^	2.6×10^−2^
	**Location: Battery Point**					
2006	2.0×10^−2^	4.9×10^−2^	4.9×10^−2^	6.4×10^−2^	1.0×10^0^	1.3×10^−2^
2007	2.4×10^−2^	6.0×10^−2^	9.8×10^−2^	5.0×10^−2^	9.6×10^−1^	1.0×10^−2^
2008	2.0×10^−2^	1.0×10^−2^	2.0×10^−2^	5.0×10^−2^	7.0×10^−1^	4.4×10^−3^
2009	4.9×10^−2^	1.0×10^−2^	2.0×10^−2^	6.0×10^−2^	7.0×10^−1^	5.6×10^−2^
2010	2.0×10^−2^	1.1×10^−2^	7.5×10^−2^	8.9×10^−2^	7.1×10^−1^	3.4×10^−3^
2011	5.2×10^−2^	1.9×10^−2^	1.5×10^−1^	9.0×10^−2^	8.5×10^−1^	5.1×10^−3^
2012	3.1×10^−2^	3.3×10^−2^	3.7×10^−2^	9.0×10^−2^	7.0×10^−1^	1.1×10^−2^
**Average**	3.1×10^−2^	2.7×10^−2^	4.5×10^−2^	7.0×10^−2^	8.0×10^−1^	2.1×10^−2^

The fittings are displayed in Figure 4.

The model was fitted to the *Cx. pipiens* complex surveillance data using Berkeley Madonna Version 8.3.18 software to estimate the model parameters. In the data fitting, we incorporated the actual insecticide treatment schedules reported by the BCMC for each location. Estimated values were established through the best nonlinear least squares fit of the model for the surveillance data, (i.e., program minimized the root mean square (RMS) between the recorded data and the analogous model predictions) (Table 4 and Table S1 in File S1).

Lower and upper bounds for the selected parameters were employed in the data fitting procedure from the previous modeling studies (listed in Table 3). We scaled the model predictions, which are for the entire neighborhood, by a factor (*p*) to compare with the mosquito surveillance data from each trap. We took the lower bound of the treatment effectiveness to be 0.7 day^−1^.The duration of the treatment effectiveness is assumed to last approximately 1 day since the ground-dispersed products are effective as contact insecticides during the night because most of the active ingredients break down within an hour after sunlight exposure.

## Results

### Collection and identification of mosquitoes

The *Cx. pipiens* complex represented 95.1% of all mosquito species collected and identified in the EVS trap located at Sams Point from 2006 to 2012 (Table 5). For the Battery Point site, the *Cx. pipiens* complex signified 86.8% of the total collections during the same 7 years (Table 6).

**Table 5:** Summary of adult female mosquitoes (with mean females per trap night) collected in an EVS trap located at Sams Point neighborhood in Beaufort County, SC from 2006–2012.

Mosquito Species	2006	2007	2008	2009	2010	2011	2012	Totals	% Totals
*Aedes albopictus*		4 (0.08)	2 (0.04)		2 (0.04)		17 (0.33)	25	0.59
*Aedes taeniorhynchus*	18 (0.35)	4 (0.08)	6 (0.12)	4 (0.08)	55 (1.06)	56 (1.08)	16 (0.31)	159	3.73
*Aedes vexans*							1 (0.02)	1	0.02
*Culex pipiens* complex	288 (5.54)	1,409 (27.10)	1,019 (19.60)	498 (9.58)	470 (9.04)	128 (2.46)	236 (4.54)	4,048	95.05
*Culex restuans*		2 (0.04)	7 (0.13)				1 (0.02)	10	0.23
*Culex salinarius*			2 (0.04)		1 (0.02)		6 (0.12)	9	0.21
*Culex territans*	2 (0.04)							2	0.05
*Uranotaenia sapphirina*						5 (0.10)		5	0.12
**Totals**	308	1,419	1,036	502	528	189	277	4,259	100.00

We fitted the model to the *Culex pipiens* complex surveillance data from both traps separately during 2006–2012.

**Table 6:** Summary of adult mosquitoes (with mean females per trap night) collected in an EVS trap located at Battery Point neighborhood in Beaufort County, SC from 2006–2012.

Mosquito Species	2006	2007	2008	2009	2010	2011	2012	Totals	% Totals
*Aedes albopictus*	3 (0.06)	18 (0.35)	8 (0.15)	4 (0.08)	5 (0.10)	4 (0.08)		42	0.93
*Aedes taeniorhynchus*		2 (0.04)	1 (0.02)		2 (0.04)	5 (0.10)	3 (0.06)	13	0.29
*Aedes vexans*	16 (0.31)	6 (0.12)	19 (0.37)	2 (0.04)	4 (0.08)	38 (0.73)	20 (0.38)	105	2.34
*Anopheles crucians*	3 (0.06)					1 (0.02)		4	0.09
*Culex erraticus*				1 (0.02)				1	0.02
*Culex nigripalpus*	8 (0.15)	3 (0.06)	5 (0.10)	13 (0.25)				29	0.65
*Culex pipiens* complex	415 (7.98)	735 (14.13)	534 (10.27)	728 (14.00)	547 (10.52)	442 (8.50)	498 (9.58)	3,899	86.80
*Culex restuans*	35 (0.67)	17 (0.33)	70 (1.35)	38 (0.73)		16 (0.31)	9 (0.17)	185	4.12
*Culex salinarius*	18 (0.35)	8 (0.15)	163 (3.13)	6 (0.12)	3 (0.06)		6 (0.12)	204	4.54
*Culex territans*	1 (0.02)		4 (0.08)					5	0.11
*Uranotaenia sapphirina*		1 (0.02)	2 (0.04)		2 (0.04)			5	0.11
**Totals**	499	790	806	792	563	506	536	4,492	100.00

We fitted the model to the *Culex pipiens* complex surveillance data from both traps separately during 2006–2012.

### Overview of the comparison with surveillance data and numerical simulations

Our data fitting results suggest declines in the number of mosquitoes after insecticide treatments, which agree with the trend of the majority of the surveillance data from both trap locations in the absence of WNV infection (Figure 4). The best-fit parameter estimates are listed in Table 4 for both trap locations separately for each year from 2006 to 2012. Root Mean Square (RMS) for the best fit of the model to the surveillance data resulted in the highest values for years 2008 and 2009 (see Table S1 in File S1) and in the lowest values for years 2006, 2011, and 2012 for both trap locations. However, due to the low numbers of mosquitoes in the Sams Point trap in 2012, our model did not capture a minor increase of mosquitoes in August-September (Figure 4). We evaluated various treatment scenarios based on the obtained parameter estimates (Figures 5 and 6). We used the best-fit parameter estimates in the model with the WNV infection, to predict the changes of human, mosquito, and bird populations during a WNV outbreak (Figure 7). Further, we conducted additional sensitivity analysis of the model parameters in Figure 8 and Figures S1–S4 in File S1.

**Figure 5:** Effectiveness of various treatment scenarios predicted by the model in the absence of the WNV infection. Demonstration of how various insecticide applications impact the adult mosquito (A and C) and larval populations (B and D). Dates of the insecticide treatments (A and B) and treatment effectiveness were varied (C and D) as indicated in the legends in each figure. The remaining parameter estimates were taken from the Tables 3 and 4 (best-fit parameter values are taken for the year 2006 from Sams Point trap location).

**Figure 6:** Sensitivity test of the predicted adult mosquito population to the model parameter representing treatment effectiveness in the absence of the WNV infection in the model. Contour plot of the adult mosquito populations as a function of the treatment effectiveness (*s*) versus time. The remaining parameters were fixed and chosen from the Tables 3 and 4 (best-fit parameter values are taken for the year 2006 from Sams Point trap location).

**Figure 7:** Model predictions of the mosquito, bird, and human populations in the presence of the WNV infection. The changes of mosquito (A–C), bird (D–F), and human (G–I) populations predicted by model (equations are listed in the Appendix S1 in File S1). The insecticide treatments scenarios, non-treatment (A, D, and G), biweekly (B, E, and H), and weekly (C, F, and I) are represented in each column. Model variables and parameter values are given in Tables 2–4 (best-fit parameter values are taken for the year 2006 from Sams Point trap location).

**Figure 8:** Sensitivity test of the predicted basic reproductive ratio to the selected model parameters. The basic reproductive ratio (ℜ_0_) as the function of the mosquito biting rate per day (*β*) and adult mosquito death rate per day (*δ_M_*). The remaining parameters in the formula are taken from the Tables 3 and 4 (best-fit parameter values are taken for the year 2006 from Sams Point trap location). The ratio formula and its derivation are provided in the Appendix S2 in File S1.

### Declines in the number of mosquitoes after insecticide treatments

According to our modeling predictions, the adulticide treatments produced significant reductions in the *Cx. pipiens* complex populations in specific neighborhoods (Figure 4). However, the abatement outcomes were effective for about one day and then the mosquito populations rebounded rapidly after the treatment became ineffective (Figure 4–6).

### Insecticide treatment scenarios

Our model shows that the number of larval and adult *Culex pipiens* complex vary as we change the frequency of adulticide applications between every 1, 2, and 4 weeks (Figure 5A and B). Insecticide applied every 2 and 4 weeks results in a higher number of larval and adult mosquitoes than the weekly abatement scenario. Our results suggest that two months of weekly insecticide treatments will suppress the larval and adult mosquito populations to minor (acceptable) levels (Figure 5A and B). When the mosquito mortality due to the treatment is decreased from 0.7 day^-1^ to 0.4 day^-1^ or 0.2 day^-1^, the vector populations are not as effectively controlled (Figure 5C and D). In particular, a mosquito mortality of 0.2 day^-1^ will result in approximately 3.5 times larger mosquito populations than the mortality of 0.7 day^-1^ (Figure 5C). The contour plot (Figure 6) for treatment effectiveness varying from 0–1 day^-1^ in which the adult mosquito population is shown as a function of the treatment effectiveness versus time provides a greater detail on the mosquito mortality needed to reduce the mosquito populations to the specific levels.

### Control strategies during a WNV outbreak

In the absence of control, the number of mosquitoes remains elevated throughout the summer (Figure 7A). In particular, the number of infected mosquitoes quickly rises to a peak about a month after the beginning of the WNV infection (Figure 7A). When the biweekly insecticide treatment is applied, the number of susceptible and infectious vectors decreases significantly after each treatment (Figure 7B). The number of infectious mosquitoes is considerably reduced during the months of June–September and the population peak is approximately 5 times lower than without insecticide control (Figure 7B). However, more frequent weekly treatments result in an insignificant number of infectious mosquitoes (Figure 7C). The total number of vectors declines to an insignificant level in August and September, only two months after the start of the weekly treatments (Figure 7C). This scenario creates a minor number of disease cases (Figure 7F and I).

Our model predicts that the number of WNV fever cases will reach a peak in the mid-July in the non- insecticide treatment scenario (Figure 7G). The significant difference in the non- treatment versus biweekly application is the number of individuals with WNV fever and time of their amplification. The number of WNV fever cases is delayed by approximately 1.5 weeks and decreased by approximately a factor of 1.5. The number of neuroinvasive cases is low in the non-treatment and biweekly application and it is negligible when a weekly treatment is applied (Figure 7G–I).

### Dead birds as disease indicators

The majority of people infected with WNV are asymptomatic or have flu-like symptoms [1]. Thus, it is difficult to detect a WNV disease outbreak based on the infrequent examination of these individuals by health care providers. However, an indication of a WNV disease outbreak may become obvious after numerous dead birds are discovered in a community. Residents can submit and/or report dead birds to the local and/or state government health department or a similar agency that monitors WNV activity. For instance, South Carolina Department of Health and Environmental Control (SCDHEC) requests the submission of a freshly dead blue jay (*Cyanocitta cristata* Linnaeus), house finch (*Haemorhous mexicanus* Muller), American crow (*Corvus brachyrhynchos* Brehm), house sparrow (*Passer domesticus* Linnaeus), and/or fish crow (*Corvus ossifragus* Wilson) from mid-March to the end of November [5]. Our modeling predictions indicate that such an occurrence of dead birds becomes noticeable in mid-June and reaches high numbers at the beginning of July in the absence of treatments (Figure 7D) and in the beginning of August when the biweekly treatments are applied (Figure 7E).

### Basic Reproductive Number

The basic reproductive number (ℜ_0_) for the model is given by (see Appendix S2 in File S1 for derivation): 


Similarly to [37], the first and second factors under the square root correspond to the number of secondary bird infections caused by a single infectious mosquito and the probability that the blood meal will be from a susceptible bird. The third factor denotes the number of secondary mosquito infections caused by one infected bird. The basic reproductive number does not depend on the secondary human infections because humans cannot infect mosquitoes with WNV. However, ℜ_0_ depends on the total blood supply (*N_Total_*) evaluated at the disease free equilibrium, which consists of the populations of birds and humans (). If ℜ_0_ is above the threshold value of 1, a disease outbreak is possible. The goal of mosquito abatement is to lower ℜ_0_ to a value below 1. In particular, ℜ_0_ depends on the mosquito death rate (*δ_M_*) and the mosquito biting rate per day (*β*), which can impact the value of ℜ_0_. For the death rate value of 0.15 day^−1^ and for the mosquito biting rate per day of 3, we estimated ℜ_0_ to be 3.02, which suggest a rapid spread of WNV. A higher death rate and a lower biting rate result in much lower ℜ_0_. In particular, the death rate of ≥0.45 day^−1^ and the biting rates ranging from 1 to 4, will decrease ℜ_0_ to below the threshold value of 1, which will prevent a WNV outbreak (Table 7). Our model predicts ℜ_0_ to decline below the threshold value when the mosquito biting rate per day is 1 and the mosquito death rate is>1.15 day^−1^ (Table 7 and Figure 8). Also, increasing the mosquito death rate to 0.35 day^−1^ and decreasing the mosquito biting rate per day to below 4 results in a ratio below 1. Various scenarios that decrease the ratio to below the threshold value and increase the probability to control the disease are summarized in Table 7 and Figure 8.

**Table 7:** Sensitivity test of the predicted basic reproductive ratio to the mosquito biting rate and the death rate of the susceptible adult mosquitoes.

	*δ_M_* = 0.15	*δ_M_* = 0.20	*δ_M_* = 0.25	*δ_M_* = 0.30	*δ_M_* = 0.35	*δ_M_* = 0.40	*δ_M_* = 0.45	*δ_M_* = 0.50
***β*** ** = 1**	1.007	0.689	0.511	0.400	0.322	0.267	0.226	0.195
***β*** ** = 2**	2.013	1.379	1.021	0.796	0.643	0.533	0.452	0.340
***β*** ** = 3**	3.020	2.068	1.532	1.194	0.965	0.801	0.679	0.585
***β*** ** = 4**	4.027	2.757	2.042	1.592	1.286	1.068	0.905	0.780

The impact of varying mosquito biting rate (*β*) and their death rate per day (*δ_M_*) on the ratio, given by the formula:  (see Appendix S2 in File S1 for derivation). The remaining parameter values in the formula are taken from the Tables 3 and 4 (best-fit parameter values are taken for the year 2006 from Sams Point trap location). The parameter definitions and units are listed in Table 3.

### Sensitivity tests

We also conducted sensitivity tests of the model parameters on the larval and adult mosquito populations (Figures S1 and S2 in File S1). We varied the parameters (described in each figure legend); specifically, we examined the upper and lower bounds of the parameters and their means (listed in Table 3). The remaining parameters were fixed at the mean of the upper and lower bounds. The variations in the initial number of larvae (*L_0_*) and adults (*M_0_*) show that these values increased proportionally with the final set point of the vector populations (Figure S1 in File S1). Sensitivity analysis of the maturation (*m*), birth (*b*), larval mosquito death (*δ_L_*), and adult mosquito death (*δ_M_*) rates on the resulting larval and adult mosquito populations show the mean values of these parameters maintain a consistent level of mosquito populations (Figure S2 in File S1). Lower bound parameter values of *m* and *b* cause the decline of these populations whereas upper bound estimates result in an increase. Conversely, lower bound parameter values of *δ_L_* and *δ_M_* cause the increase of these populations whereas upper bound estimates result in a decrease. This outcome suggests that decreasing *m* and/or *b* and/or increasing *δ_L_* and/or *δ_M_* will reduce the mosquito populations. For example, residents and visitors could support mosquito abatement efforts by removing *Cx. pipiens* complex breeding sites, such as water-filled containers, thus increasing *δ_L_*, which will result in a decrease of the larvae and, subsequently, the adult mosquito populations.

In addition, we have also conducted sensitivity tests of predicted infected mosquitoes (*M_I_*), infected birds (*B_I_*), and humans with WNV fever (*H_F_*) populations to the initial values in the model with WNV infection (Figure S3 in File S1) and sensitivity tests of predicted infected mosquitoes (*M_I_*), infected birds (*B_I_*), dead birds due to the infection with WNV (*B_D_*), humans with WNV fever (*H_F_*) populations to the mosquito biting rate per day (*β*) (Figure S4 in File S1). These sensitivity tests depict the differences in the time and height of the infection peak as the initial conditions and the mosquito biting rate are varied.

## Discussion

Mosquito surveillance data was evaluated for a specific mosquito trap used to collect *Cx. pipiens* complex mosquitoes, primary vectors of WNV in regions of the U.S. [6]. While comparison to the field data is vital to estimate the effectiveness of various mosquito control strategies, previous modeling efforts rarely utilized surveillance data to estimate the parameters and validate the models. Our modeling predictions and the trend of the majority of the surveillance data depict declines in the number of mosquitoes after each insecticide treatment (Figure 4). The data and curves generated by our model show significant declines in the number of mosquitoes when insecticide treatments are applied; however, the vector populations rebound rapidly (Figure 4–6). These results suggest that frequent applications of public health insecticides are necessary to control adult vectors and, ultimately, the spread of WNV. As part of a multidisciplinary approach before and during a WNV outbreak, this control strategy should be supplemented by: 1) source reduction or the elimination of breeding sites, 2) treatment of catch basins and other suitable breeding sites, and 3) initiation of community outreach activities.

Through the data fitting procedure, we obtained parameter estimates (Table 4) that enabled us to attain a more reliable evaluation of the treatment effectiveness and predictions during a WNV outbreak at a specific location (Figure 7). We identified the treatment scenarios necessary to control WNV transmission and conducted sensitivity analysis of the selected model parameters (Figures 5–8 and Figures S1–S4 in File S1). Our model predicts a minimal number of mosquitoes and, subsequently, negligible WNV transmission when weekly insecticide treatments are conducted (Figure 7C, F, and I). Further, we investigated the impact of mosquito biting rate and their death rate on the basic reproductive ratio (Table 7 and Figure 8). We concluded that lower values of mosquito biting rate and higher mosquito death rate results in lower values of ℜ_0_ (Table 7 and Figure 8) and if we can lower it enough to achieve ℜ_0_<1, then an epidemic can be avoided.

We also demonstrated that in the biweekly treatments and non-treatment scenarios an increase in the number of dead birds would be observed, which would be an indicator of a WNV outbreak (Figure 7D and E). Not all birds have the same mortality rate due to WNV infection. For example, an experimental study reported that the common grackle (*Quiscalus quiscula* Linnaeus) had a mortality rate of 33% in contrast to the American crow, red-billed gull (*Larus scopulinus* Forster), and the house finch, which depicted nearly 100% mortality rates [43]. A future modeling study could assess more classes of birds depending on their susceptibility and morality due the infection. However, more data is necessary to adequately estimate the unknown parameters in a more complex model with these features.

A large occurrence of American crow die-offs preceded the 1999 laboratory confirmation of WNV among various bird species in New York [44]. Also, abnormal bird deaths (primarily American crows) were observed in 2003 at Riverside, CA and nearby areas prior to a WNV outbreak [45]. The number of birds reported by the second month of the outbreak was about 5,000. This number represented a small portion of the bird mortalities because of the discontinued use of the residential hotline when dead bird sightings became common [45]. Other areasin California (Kern and Los Angeles counties) reported bird die offs during the summer of 2004 [46].

A recent study reported that the blood feeding behavior of *Cx. quinquefasciatus* significantly shifted with the change of season [47]. While another study noted that the feeding preference varied completely with location [48]. Further, information of the local regional preference is necessary to obtain reasonable estimates of the host feeding preference percentages. Although *Cx. quinquefasciatus* may have a preferred host for blood feeding, however availability of hosts is a key factor for an ultimate choice. We have added a variation of the model that includes feeding preferences in the Supplementary Materials (see Appendix S3 in File S1).

A limitation in our study is the impact of various natural factors, such as the seasonality of the vector populations. Many factors affect the rate at which mosquitoes reproduce, including larval rearing conditions, adult size, age, and the quality and quantity of the blood meal [49]. In a recent study of larval abundance in stormwater catch basins, low precipitation and high mean temperature were associated with high larval abundance in urban and suburban areas [50]. A study of spatiotemporal dynamics of the spread of WNV demonstrated a key role of the temperature on the seasonality and emergence of WNV [51]. Therefore, we have considered only a short duration (June–September) for multiple years in our study to avoid the dependence of the model on the aforementioned parameters.

Another limitation of the study is the treatment effectiveness that may vary with time and space. The insecticide treatment in our study is very effective for a short period of time and we have reviewed data from two locations in which treatments were applied throughout the neighborhoods on specific dates. Such changes in the treatments may be considered upon availability of other data.

There is a need to study temperature and rain events for evaluating the development of the *Cx. pipiens* complex throughout the underground stormwater systems. In past studies, the design of underground management systems and water temperature significantly impacted the development cycles of *Culex* mosquitoes [52], [53]. Furthermore, other relationships between natural factors and mosquito populations can be reviewed by analyzing data and constructing mathematical models, which are essential to optimize control methods for a particular mosquito breeding habitat.

Surveillance strategies can be improved by increasing the frequency of samples collected throughout the year as well as increasing the number of strategically located mosquito trap sites. These changes may reduce uncertainties among the collected data and would assist to quantify the effects of inconsistent weather conditions, such as floods and droughts, on the various mosquito populations. Upon the establishment of these relationships, it would be possible to propose improved surveillance and abatement strategies to monitor and control the mosquito populations. Our modeling results support the long-standing importance of mosquito control and surveillance activities.

## Supporting Information

File S1 **Supplementary appendices, table, and figures.** **Appendix S1**, Model Equations. **Appendix S2**, Basic Reproductive Number. **Appendix S3**, Mosquito Feeding Preferences. **Table S1, Root Mean Square generated by the best fit of the model to the** ***Culex pipiens*** **complex** **surveillance data collected in EVS traps located in Sams Pont and Battery Point.** The model was fitted to the surveillance data using Berkeley Madonna Version 8.3.18 software to estimate the model parameters. Estimated values were established through the best nonlinear least squares fit of the model for the surveillance data, (i.e. program minimized the root mean square (RMS) between the recorded data and the analogous model predictions). **Figure S1, Sensitivity tests of predicted larva and adult mosquito populations to their initial values in the absence of the WNV infection in the model.** Plots illustrating the sensitivity of the initial number of larval (*L_0_*) and adult mosquitoes (*M_0_*) on the subsequent larval and adult mosquito populations, respectively. The initial condition parameter in the legend was varied while the remaining parameters were fixed and chosen from the Tables 3 and 4 (best-fit parameter values are taken for the year 2006 from the Sams Point trap location). **Figure S2, Sensitivity tests of predicted larva and adult mosquito populations to the model parameters in the absence of the WNV infection in the model.** Plots illustrating the sensitivity of the maturation (*m*), birth (*b*), larval mosquito death (*δ_L_*), and adult mosquito (*δ_M_*) rates on the subsequent larval and adult mosquito populations, respectively. The parameter in the legend was varied while the remaining parameters were fixed and chosen from the Tables 3 and 4 (best-fit parameter values are taken for the year 2006 from the Sams Point trap location). **Figure S3, Sensitivity tests of predicted infectious mosquitoes, infectious birds, and humans with WNV fever populations to the initial values in the model with WNV infection.** Plots illustrating the sensitivity of the initial susceptible populations of female adult mosquitoes (*M_0_*), birds (*B_0_*), and humans (*N*) on the infected mosquitoes (*M_I_*), infectious birds (*B_I_*), and humans with WNV fever (*H_F_*) populations. The initial condition parameter in the legend was varied while the remaining parameters were fixed and chosen from the Tables 3 and 4 (best-fit parameter values are taken for the year 2006 from the Sams Point trap location). **Figure S4, Sensitivity tests of predicted infectious mosquitoes, infectious birds, dead birds due to the infection with WNV, humans with WNV fever populations to the mosquito biting rate per day.** Plots illustrating the sensitivity of the mosquito biting rate per day (*β*) on the infectious mosquitoes (*M_I_*), infectious birds (*B_I_*), dead birds due to the infections with WNV (*B_D_*), and humans with WNV fever (*H_F_*) populations. The mosquito biting rate per day in the legend was varied while the remaining parameters were fixed and chosen from the Tables 3 and 4 (best-fit parameter values are taken for the year 2006 from the Sams Point trap location).
(DOCX)
